# MiR-373 Inhibits the Epithelial-Mesenchymal Transition of Prostatic Cancer via Targeting Runt-Related Transcription Factor 2

**DOI:** 10.1155/2021/6974225

**Published:** 2021-06-29

**Authors:** Jianyi Pang, Limei Dai, Chen Zhang, Qinglei Zhang

**Affiliations:** ^1^Department of Urology Surgery, The Affiliated Weihai Second Municipal Hospital of Qingdao University, Weihai, Shandong 264200, China; ^2^Department of Dermatology and STD, The Affiliated Weihai Second Municipal Hospital of Qingdao University, Weihai, Shandong 264200, China; ^3^Department of Urology Surgery, The Affiliated Tengzhou Central People's Hospital of Jining Medical University, Tengzhou, Shandong 277500, China

## Abstract

Prostatic cancer (PCa) is a prevalent form of malignancy based on its high associated levels of mortality and morbidity across the world. MicroRNAs (miRNAs) are significant in the advancement of prostatic cancer. The current study is aimed at exploring the potential roles of miR-373 in PCa. In turn, the study conducted a qRT-PCR test to determine the levels of mRNA. A western blot test was also executed in determining the protein level. The processes of transwell assay and wound healing were integrated in the detection of the potential for PCa cells to invade and migrate. The integration of dual luciferase reporter assay is critical in determining the levels of luciferase activity among prostatic cancer cells. Then, the results showed a net decrease of miR-373 within prostatic cancer cells and tissues. Upregulated miR-373 reduced the invasion and migration potential of PCa cells. Moreover, overexpressed miR-373 increased the levels of E-cadherin and FSP1 as epithelial cell markers. Similarly, the overregulation of miR-373 brought about the upregulation of mesenchymal markers (N-cadherin, Snail, and vimentin). The study predicted runt-related transcription factor 2 (RUNX2) to be a target of miR-373. The luciferase activity of PCa cells was decreased after the cotransfection with miR-373 mimics and RUNX2 3′ untranslated region (3′UTR) wild type (WT). Moreover, RUNX2 became upregulated in PCa cells and tissues. The upregulation of miR-373 decreased the mRNA and protein level of RUNX2. However, overexpressed RUNX2 abated the roles of miR-373 in the intrusion and migration of PCa cells and in regulating the expression of epithelial cell markers and mesenchymal markers. In short, miR-373 may regulate the EMT of PCa cells via targeting RUNX2. The miR-373/RUNX2 axis provides a therapeutic target for PCa.

## 1. Introduction

PCa, characterized with high mortality and morbidity, is one of the most malignant tumors worldwide [1, 2]. The past years saw an increase of morbidity and mortality of PCa patients [3, 4]. The PCa-related deaths in 2012 reached 300,000 [5]. Additionally, the mortality of PCa increased from 3/100,000 to 30/100,000 in Asia [6]. Although prestigious breakthroughs have been realized in the management of PCa, the overall rates of survival in PCa are still unsatisfactory. In part, the diagnosis of patients at advanced stages is responsible for the low survival rates. The average survival rate over 5 years is 90% at early stage, while it is no more than 15% at advanced metastatic stage [7]. Lymph node metastasis and bone metastasis are the main challenges in the treatment of prostate cancer [8]. Epithelial-mesenchymal transition (EMT) remodels cell-cell and cell-extracellular matrix interactions, which induces the initiation and metastasis of cancer [9]. Therefore, to suppress the metastasis of PCa may be a promising therapy for the management of PCa.

MicroRNAs (miRNAs) are small endogenous noncoding RNAs, which play a crucial role in post-transcription [10]. Besides, miRNAs degrade gene level through their potential to bind to the 3′ untranslated region (3′UTR) within the target genes [11]. Intensive bodies of evidence have reported that miRNAs participate in multiple biological processes, including proliferation, cell differentiation, invasion, apoptosis, and migration, and epithelial-mesenchymal transition [12, 13]. Moreover, the aberrant expressed miRNAs are significant in facilitating the progression and emergence of cancer, including PCa. For instance, miR-373 is downregulated in non-small cell lung cancer (NSCLC), while overexpressed miR-373 suppresses EMT of NSCLC cells [14]. Upregulated miR-373 promotes EMT of tongue squamous cell carcinoma. MiR-373 is decreased in human epithelial ovarian cancer (EOC), while its overexpression suppresses the invasion and EMT of EOC cells [15]. MiR-373 inhibits the invasion of progression of PCa [16]. However, the underlying mechanisms is still unclear.

Still, RUNX2 is firstly reported to participate in the skeletal embryogenesis. In recent years, its oncogenic properties have been attracting increasing attention. RUNX2 is involved the initiation and progression of numerous cancers [17–19]. RUNX2 acts as an oncogene and regulates the apoptosis, migration, proliferation, invasion, and ETM of malignant cells via unchecked signaling pathways [18, 19]. In PCa, overexpressed RUNX2 is associated with high-grade prostatic intraepithelial neoplasia (HGPIN), cancerous lesions, and prostate tumorigenesis [20]. However, the possible roles of RUNX2 in EMT of PCa have not been elucidated.

In this study, transwell assay and wound healing were applied to examine the implications of overexpressed miR-373 on the processes of invasion and migration among PCa cells. The concept of luciferase assay has the potential of providing novel therapeutic target and was thus used in verifying whether RUNX2 was a target of miR-373. In summary, the study was based on the purpose of investigating the potential roles of miR-373 in the EMT of PCa and the underlying molecular mechanisms.

## 2. Methods

### 2.1. Clinical Samples

Tissue samples from the PCa as well as normal tissues in adjacent locations were selected from 30 patients diagnosed with PCa. Besides, the control population entailed patients that had benign prostatic hyperplasia (BPH) during August, 2017, to January, 2019, at The Affiliated Weihai Second Municipal Hospital of Qingdao University. The samples were immediately placed at a temperature of −80°C following the surgery. Besides, the participants have not received chemotherapy or radiotherapy prior to this study. The supervision of the research was conducted by the Institutional Review Board within the sponsoring institution. However, all participants were required to sign and provide informed consent.

### 2.2. Cell Culture

The researchers purchased their cell culture from ATCC and included normal prostate epithelia cell line alongside LNCaP, and DU145. Similarly, human PCa cell lines PC3 were also sourced from the cell culture in ATCC. Cells were incubated in a basal medium with 10% concentration of FBS and Penicillin-Streptomycin at 1%. Moreover, the temperature of the incubator was controlled at 37°C with 5% CO_2_. The cells were subjected to a confluence of 80% through the process of being passaged.

### 2.3. Transfection

The transfection of PC3 cells was achieved using 50 nM of miR-373 mimics (Mimics) or miR-NC mimics (NC mimics) using Lipofectamine 2000 (Invitrogen, USA) for 48 h. pcDNA3.1 and pcDNA3.1-RUNX2 were synthesized and provided by GenePharma (Shanghai, China). The transfection of the cells was achieved using either pcDNA3.1-RUNX2 or pcDNA3.1 based on the manufacturer's protocols that use lipofectamine 2000.

### 2.4. qRT-PCR

The choice of reagent for isolating total RNA from the localized cells and tissues was TRIzol. The collected RNA was then transcribed into cDNA with PrimeScript RT kit (Takara, Japan) based on the manufacturer's instructions. The PCR was conducted using SYBR® Premix ExTaq™ II Kit (Takara, Japan) under the prescribed thermo cycling condition. Particularly, it was exposed to five minutes at 95°C, and 40 more cycles averaging 30 seconds at a temperature of 95°C. Finally, it was subjected to further cycles of 45 sec at 60°C. Then, a calculation of the expression level was made using 2^−∆∆CT^ method. In turn, U6 was regularized to the prescribed levels of miRNA and GAPDH to mRNA.

### 2.5. Western Blot

Cells or tissues were lysed. Total protein was collected with RIPA buffer (Sigma-Aldrich, USA). The concentration of the protein was calculated with BCA kit (Pierce, USA). Then, total protein was isolated with 12% SDS-PAGE. Afterwards, the protein was moved onto PVDF membranes, which was then blocked with milk that possessed nonfat attributes. The membranes would then be incubated over the night by relying on primary antibodies and being put in temperatures of 4°C in shade and then with secondary antibodies. Subsequently, the protein was visualized, and the relative protein level was calculated.

### 2.6. Wound Healing Assay

After 48 h transfection, cells became cultured with a 6-well plate (3 × 104 cells/well) overnight till the cells reached 80–90% confluency. Then, a pipette tip was applied to make a scratch. The cell movement was pictured and analyzed.

### 2.7. Transwell Assay

The cells were placed into a 24-well plate (2 × 103 cells/well) and then incubated in the upper chamber containing Matrigel and serum-free DMEM. Inherently, the bottom chamber was treated with 10% FBS. Within a day, the noninvasive cells were removed. Next, the invaded cells were corrected with 4% methanol while crystal violet was used for staining. Finally, the cells were captured before being calculated.

### 2.8. Dual Luciferase Reporter Assay

The online database across TargetScan 7.2 (https://www.targetscan.org/vert_72/) was utilized to forecast the target of miR-373. The 3′ untranslated region (3′UTR) sequences containing the potential target of miR-373 were synthesized and cloned into reporter gene plasmid vector pGL3 to build RUNX2 3′UTR wild type and RUNX2 3′UTR Mutant (MUT) plasmids. Then, the transfection of the cells is achieved using either miR-373 NC or the same variant with an accompanying Lipofectamine 2000 at 37°C with 5% CO_2_. The determination of the cell luciferase activity was consistent with the Dual-Luciferase Reporter Assay System (Promega, USA).

### 2.9. Statistical Analysis

Data collected in the study was analyzed with SPSS22.0 software and represented through calculations of mean ± standard deviation (mean ± SD). The variances between the two groups were considered using Student's *t*-test, while the variances in multigroups were evaluated with one-way ANOVA. The statistical significance was set at *P* < 0.05.

## 3. Results

### 3.1. MiR-373 Is Downregulated in PCa Tissues

qRT-PCR was executed to identify the manifestation of miR-373 in PCa tissues as well as the normal tissues adjacent to the malignant cells. As shown in Figure 1, the expression of miR-373 was downregulated in PCa tissues relative to the normal tissues in adjacent locations, thereby suggesting that miR-373 may be an antitumor miRNA in PCa.

### 3.2. MiR-373 Is Decreased in PCa Cells

In exploring the roles of miR-373 in PCa, we also detected the expression of miR-373 in PCa cells. The findings also portrayed a decrease in the volume of miR-373 in PCa cell lines, such as PC3, LNCaP, and DU145, compared with prostate epithelial cell line RWPE-1, which was more potent in PC3 (Figure 2(a)). Then, PC3 cells were used in the following experiment. Moreover, the manifestation of miR-373 in PC3 cells that were transfected with miR-373 mimics was upregulated in comparison with control populations, which suggested PC3 were successfully transfected (Figure 2(b)).

### 3.3. MiR-373 Inhibits the EMT of PCa Cells

The processes of transwell assay and wound healing were executed to test the implications of miR-373 on the intrusion and migration of PCa cells. As shown in Figure 3(a), the scratch width of the miR-373 mimics transfected cells showed no significant difference. In turn, the healing rate was significantly decreased, suggesting that miR-373 inhibited the potential for PCa cells to migrate. Moreover, the ability of PCa cells to invade is significantly inhibited when transfected with miR-373 mimics, relative to the control group (Figure 3(b)). Meanwhile, overexpressed miR-373 downregulated N-cadherin, Snail, and vimentin and upregulated E-cadherin and FSP1, suggesting miR-373 played an inhibitory role in the EMT of PCa cells (Figure 3(c)).

### 3.4. MiR-373 Directly Targets RUNX2

The research predicted RUNX2 as a target of miR-373 (https://www.targetscan.org/vert_72/). The binding locations between miR-373 and RUNX2 are shown in Figure 4(a). The findings from the luciferase assay portrayed the fact that the luciferase activity of PCa cells was transfected along with miR-373 mimics and RUNX 3′UTR WT was considerably decreased compared with NC mimics group (Figure 4(b)). The protein rates of RUNX2 were upregulated in PCa cells and tissues (Figures 4(c) and 4(d)). However, the mRNA of RUNX2 was also downregulated following its transfection with miR-373 mimics, which was paralleled with the protein level (Figures 4(e) and 4(f)).

### 3.5. Overexpressed RUNX2 Alleviates Inhibition of EMT Induced by MiR-373 Mimics in PCa

Rescue assay was performed to examine the roles of RUNX2 in the EMT of PCa cells. As shown in Figures 5(a) and 5(b), upregulated miR-373 reduced the potential for invasion and migration among PCa cells when compared with NC mimics, which was reversed by the overexpression of RUNX2. Moreover, the regulatory role of miR-373 in the depiction of EMT-related genes (such as N-cadherin, Snail, vimentin, E-cadherin and FSP1) was alleviated by RUNX2, where upregulated RUNX2 alleviated the effects of miR-373 on the EMT of PCa cells (Figure 5(c)).

## 4. Discussion

Augmenting bodies of evidence have revealed miRNAs have a significant role in the initiation and sustenance of PCa [16, 21, 22]. The aberrant expressed miRNAs suppress the identified tumors in PCa. For instance, downregulated miR-129-3p is associated with TNM staging, differentiation of PCA tumor, and lymph node metastasis, while its overexpression inhibited the spread and invasion of PCa cells [23]. miR-601 functions as an oncogene in PCa. As such, it alleviates the potential for migration, invasion, and progression of PCa cells [24]. Meanwhile, Qiu et al. demonstrated that the downregulation of miR-373-3p induces the metastasis of PCa, and the silence of testicular nuclear receptor 4 (TR4) or the upregulation of miR-373-3p may be a likely target for PCa [25]. There was a reduction of miR-373 in PCa cells and tissues, thereby suggesting that miR-373 serves as an antitumor gene in PCa. These results are consistent with Qiu et al.'s study [25]. However, the possible mechanism that miR-373 regulated the progression of PCa is still unclear.

Epithelial-mesenchymal transition (EMT) is a complicated progress involved in the metastasis, stemness, and drug resistance of PCa [26]. EMT progresses with the loss of epithelial functions and acquisition of mesenchymal features [27]. This degradation from cuboidal to spindle-shaped in cell phenotype is accompanied with the downregulation of epithelial cell markers (E-cadherin, occludins, and FSP1). Similarly, mesenchymal markers such as vimentin and N-cadherin have been upregulated and further activating the master regulator of EMT, such as Snail and Twist [28, 29]. Thence, to explore the expected molecular mechanisms involved in the EMT of PCa cells to inhibit the metastasis is of vital importance. Still, miRNAs contribute to the initiation and sustenance of cancers via regulating multiple biological processes including EMT [12, 13]. In this study, upregulated miR-373 reduced the potential for invasion and migration among PCa cells. Moreover, its overexpression decreased the expression of mesenchymal markers (vimentin and N-cadherin) and the master regulator of EMT (Snail) and enhanced the manifestation of epithelial cell markers (E-cadherin and FSP1), which suggested the upregulation of miR-373 repressed the loss of epithelial functions and acquirement of mesenchymal features, and therefore inhibited the progression of EMT of PCa cells. However, the underlying mechanisms is still unknown.

miRNAs regulate biological functions through provision of bonds to the 3′UTR of the identified genes [11]. Runt-related transcription factor 2 (RUNX2) was predicted and proved to be a target of miR-373. Increasing studies have reported the upregulation of RUNX2 derived from epithelial tissues induces the progression of multitype cancers [17–19]. RUNX2, as a linage specific transcription factor, collectively participates in EMT and promotes the maturation of mesenchymal markers via interacting with specific pathways related to these pathophysiological processes [30, 31]. In PCa, the abnormal upregulation of RUNX2 contributes to EMT of PCa cells and PCa to bone metastasis [32]. In the current study, RUNX3 was upregulated in PCa cells and tissues. Interestingly, overexpressed RUNX2 reversed the alleviation of PCa invasion and migration and abrogated the upregulation of epithelial markers and the downregulation of mesenchymal markers in induced by miR-373. The findings suggested the regulatory role of miR-373 in PCa EMT was alleviated by RUNX2. Therefore, miR-373 may inhibit the EMT of PCa cells via targeting RUNX2.

In conclusion, miR-373 was downregulated in PCa cells and tissues. Overexpressed miR-373 inhibited the transition from epithelial to mesenchymal state for PCa through targeting PCa. In turn, the inhibition of this transition provides a significant strategy in the treatment of prostate cancer (PCa).

However, the present study has some limitations. Firstly, more patients are needed to make the results more convincing. Secondly, a miRNA may have more than one target, which may be targeted by various miRNAs. Therefore, the underlying mechanisms that miR-373 regulates the EMT of PCa need further research. Furthermore, this study needs to be combined with other hospitals for multicenter research in the future to promote the basic treatment of liver cancer.

## Figures and Tables

**Figure 1:** MiR-373 was downregulated in PCa tissues. The evidence of miR-373 was identified by qRT-PCR. ^∗∗^*P*<0.01 vs. normal tissues.

**Figure 2:** MiR-373 is decreased in PCa cells. (a) The manifestation of miR-373 in PCa cells. (b) The transfection efficacy of PCa cells determined by qRT-PCR. ^∗∗^*P*<0.01 vs. RWPE-1 cells or even control populations.

**Figure 3:** MiR-373 inhibits the EMT of PCa cells. (a) The potential for migration in PCa cells determined by wound healing assay. (b) The potential for invasion in PCa cells examined through transwell assay. (c) The protein level of N-cadherin, Snail, and vimentin and E-cadherin and FSP1 measured by western blot. ^∗∗^*P* < 0.01 vs. control group.

**Figure 4:** MiR-373 directly targets RUNX2. (a) The binding sites of miR-373 on RUNX2. (b) The activity of luciferase within PCa cells was established through Dual luciferase reporter assay. (c) The levels of protein in RUNX2 of PCa tissues determined by western blot. (d) The levels of protein of RUNX2 in PCa cells were identified by western blot. (e) The level of mRNA of RUNX2 in PCa cells calculated with qRT-PCR. (f) The level of protein in RUNX2 measured by western blot. ^∗∗^*P* < 0.01 vs. normal tissues, RWPE-1 cells, or control group.

**Figure 5:** Overexpressed RUNX2 alleviates inhibition of EMT induced by miR-373 mimics in PCa. (a) The potential for migration in PCa cells is established through wound healing assay after miR-373 mimics transfection and pcDNA3.1 RUNX2. (b) The potential for invasion of PCa cells examined by transwell assay after miR-373 mimics transfection and pcDNA3.1 RUNX2. (c) The protein level of N-cadherin, Snail, and vimentin and E-cadherin and FSP1 determined by western blot after miR-373 mimics transfection and/or pcDNA3.1 RUNX2. ^∗^*P* < 0.01 vs. control group. ^##^*P* < 0.01 vs. miR-373 mimics group.

## Data Availability

The simulation experiment data used to support the findings of this study are available from the corresponding author upon request.
